The article "Multidimensional Collaborative Management of Environment and Economy in the Internet-of-Things Environment" was retracted in 2023. Reasons: unreliable results or conclusions; concerns about the data; concerns about the peer review; concerns about the citations.

# Multidimensional Collaborative Management of Environment and Economy in the Internet-of-Things Environment

**DOI:** 10.1155/2022/5491677

**Published:** 2022-05-31

**Authors:** Rui Yu, Ling Han

**Affiliations:** ^1^School of Economics and Management, Xi'an University of Technology, Xi'an, Shaanxi 710054, China; ^2^Xi'an Medical University, Xi'an, Shaanxi Province 710021, China

## Abstract

In this study, multidimensional collaborative management of the modern environmental economy is proposed for strategic management, distribution management, service quality management, and warehouse management, which the modern environmental economy enterprises face under the internet-of-things environment. This study studies the law of multidimensional coordination of environmental economy and puts forward the classification of the modern multidimensional coordination of environmental economy. The multidimensional synergetic-order parameter equation of the modern environmental economic system is constructed, and the information synergy is the order parameter of the environmental economic system by accurate elimination method, and the fluctuation and balance of the environmental economic system are accurately controlled by the order parameter. By using structural equation modeling and other quantitative research methods, the corresponding planning and decision-making mathematical model is established, which provides relevant support for the realization of informatization and intelligentization of multidimensional collaborative management of the environment and economy. An incentive internal management collaboration model based on right of entry is proposed. Aiming at the problem of multidimensional environmental economic management coordination, a dynamic multidimensional environmental economic coordination management algorithm was designed by using the decomposition method, and the effectiveness of the algorithm was verified by numerical experiments.

## 1. Introduction

The modern environmental economic industry is a modern service industry integrating transportation, storage, freight forwarding, and information industries. It involves many fields and plays a very important role in promoting production and stimulating domestic demand. With the rapid expansion of industrial base and the rise of consumer market, environmental economic industry is in a stage of rapid development [1]. As a crucial part of economic development, environmental economic industry has been attached great importance to by decision-making departments. Internet technology brings to the environment economic industry informatization, automation, integration of environmental economics, and management, process monitoring technology not only bring to enterprise environment to promote the efficiency of the economy and cost control ability to strengthen environmental and economic benefits, and overall improve the informatization level of enterprises and related areas, so as to achieve the purpose of driving the development of the industry.

The article "Multidimensional Collaborative Management of Environment and Economy in the Internet-of-Things Environment" was retracted in 2023. Reasons: unreliable results or conclusions; concerns about the data; concerns about the peer review; concerns about the citations.

The efficiency of resource allocation is closely linked with the structure of resource allocation, and the two are inseparable [2, 3]. The so-called efficiency of resource allocation refers to the choice of opportunities among various possible uses of resources, focusing on the relationship between cost and income of resources. The structure of resource allocation is an opportunity choice reflected in regions, industries, enterprises, and products. Economic activity main body in the normal economic activities and possible economic development goal will require different types at different times, different locations, and different amounts of resources and make the free flow of resources reasonable, and eventually form satisfies the requirement of economic activity and the move to conform to the goal of economic development and reasonable allocation of resource structure. However, in a certain period of time, the total amount of economic resources available for social distribution is limited to a certain extent, and it takes a long time for economic resources to reach a certain accumulation [4], so it is difficult to develop advantageous enterprises and industries by solely relying on incremental resource accumulation in theory. Another way is in the stock of resources, to speed up the stock of flow velocity and frequency of resources, and to increase the intensity of product structure and industrial structure adjustment, to a large number of stock resources from disadvantaged businesses and industry transfer out [5], both to revitalize the stock resources; idle underutilized resources' economic potential was exhumed. In addition, a large amount of capital can be gathered in a short period of time to rapidly develop competitive enterprises and industries and improve the utilization efficiency of economic resources in the whole society.

Economic system is a self-organizing coordination system, and competition and coordination are the contradictory unity of self-organizing existence and development of economic system [6]. It is reasonable to use the capability theory to explain the economic element of the combination of productive function and transactional function. The theoretical framework of “synergy capacity, resource allocation, and economic performance” was constructed to analyze the problems of multidimensional environmental economic synergy economy [6], and it is believed that synergetic capacity is the fundamental factor determining the existence and development of multidimensional environmental economy, and also the fundamental factor determining its economic performance. Scale economy generally refers to the economic phenomenon that unit product costs are reduced and benefits are improved due to the expansion of production scale of economic organizations. In other words, people choose and scientifically control the production scale according to the changes in the input amount of production factors and their combination mode, so as to change the production batch [7] and achieve increased production or savings. According to the general view of economists, scale economy refers to the decrease in unit product cost caused by the increase in various input factors and the expansion of production scale under the premise of unchanged technological conditions. It is manifested by increasing returns to scale, that is, after the production scale is expanded, the increase in returns is greater than the increase in scale [8].

The article "Multidimensional Collaborative Management of Environment and Economy in the Internet-of-Things Environment" was retracted in 2023. Reasons: unreliable results or conclusions; concerns about the data; concerns about the peer review; concerns about the citations.

In order to make up for the imperfection of cooperative operation mechanism of environmental economic enterprises, the order parameter equation of the modern environmental economic system is established and solved by the quantitative analysis method. It is concluded that information synergy is the order parameter affecting system synergy.

## 2. Related Works

Existing research divides management mechanism into three types, namely, formation mechanism, implementation mechanism, and constraint mechanism. As the first step of management synergy mechanism, formation mechanism is the foundation and prerequisite of management synergy mechanism. The realization mechanism is based on the formation mechanism, which is regulated by a series of links to achieve synergetic effect. As a guarantee constraint mechanism, it plays a protective role in the whole synergy process [9, 10]. This study studies the conditions for realizing management synergy [11] and analyzes the conditions for enterprises to realize synergy and create benefits of synergy. One is the confidence and determination of enterprise managers; second, the team's incentive mechanism; and third, effective internal communication. At the same time, some scholars took multinational corporations as an example to study how enterprises can achieve coordination in expanding global business in the changing environment.

There are many ways for enterprises to achieve synergistic benefits, such as through interenterprise business behavior, just sharing, and information flow. [12]. However, it does not mean that these methods can completely solve the problem of synergy. The root cause is that sharing is limited, and only enterprises with innovative ability can truly achieve the synergetic effect. We study on the constraint mechanism of management coordination. As an important means to realize management collaboration, the constraint mechanism of management collaboration plays an important role in the whole process of management collaboration, which can be specifically divided into constraints in the formation of management collaboration and constraints in the realization of management [13]. From regional environment has made an analysis of the synergy of economic cluster [14], and their operating environment of the regional environmental economic system innovation and mode of operation, to improve the microeconomic entity, enhance the transformation of the traditional economy to the modern environment, and play a very important role, in the process of promoting the development of regional economy, with high efficiency, the direction of the sustainable development. At the same time, the innovation of regional environmental economic system pays more attention to the coordination of the system as a whole, not only to the correlation between the subsystems in time and space. The regional environmental economy itself has complexity. From the perspective of semantic web services, the collaborative environmental economy and integration technology are analyzed [15, 16].

The article "Multidimensional Collaborative Management of Environment and Economy in the Internet-of-Things Environment" was retracted in 2023. Reasons: unreliable results or conclusions; concerns about the data; concerns about the peer review; concerns about the citations.

With the advent of the new century, the voice of a coordinated environmental economy is more intense. Through the internet, enterprises can synchronize and coordinate various business activities, reduce enterprise costs, and improve enterprise profits and performance, and the network has made outstanding contributions. In this study, the structure chart of service-oriented collaborative environmental economic system is put forward. It is concluded that in dynamic alliance, the first step of business cooperation is to determine the appropriate manufacturer according to the customer demand and the quotation of the other party, and then access the order service provided by the manufacturer. After the firm is determined, the collaboration flow is basically the same as that of the fixed enterprise alliance. The same is true when manufacturers choose modern environmental economic companies. Quantitative studies on the level of system collaboration, the way of system collaboration, and the construction of collaborative system are lacking [17, 18]. Under the preparation of order parameters, the original disordered regional environmental economic industry absorption forms a new spatial and temporal cooperative state, and the regional environmental economic industry cluster appears. With the change in external environment and the interference of other factors, the industrialization cluster of regional environmental economy produces self-organization and becomes a new collaborative network of regional environmental economic innovation. The demands of remanufacturing environmental economic system are met based on real-time docking, optimal allocation of resources, reasonable equipment scheduling, the service needs of the fast integration, by building a IoT of remanufacturing closed-loop multidimensional environmental [19] economic information service system, to achieve the closed-loop multidimensional environmental economic informatization, automation, intelligence, and value chain management. By establishing the intelligent assembly system model of integrated control based on the internet of things, issues such as token routing and system deadlock in the digestion system were studied [20]. The classification method of manufacturing resources in the internet-of-things environment was proposed, and the relevant model and system framework of IoT manufacturing were constructed based on the need of realizing interconnected perception and information integration. Based on the concept of internet of things and demand model, information model, security model, communication model, function model, and deployment model, the IoT architecture framework and the relevant network address are put forward, semantic and intelligent operation, and the big data, and so on, and key theory and technology research, and technology standardization and other issues are discussed in this study. The research on synergetic science in the field of environmental economy is scattered, and there is no systematic and scientific unified standard. There is a lack of theory to guide the application of practice. There are few research studies on the synergy of environmental economic system, most of which focus on the macroperspective of multidimensional environmental economic synergy, regional environmental economic enterprise synergy, and so on, and there are few research studies on the multidimensional demand of synergy from the environmental economic system itself. In the analysis of coordination mechanism and system coordination, there are superficial and general problems, and the equilibrium state of environmental economic system is not analyzed from the angle of coordination theory.

The article "Multidimensional Collaborative Management of Environment and Economy in the Internet-of-Things Environment" was retracted in 2023. Reasons: unreliable results or conclusions; concerns about the data; concerns about the peer review; concerns about the citations.

Based on the research status at home and abroad and the deficiency of multidimensional collaborative management in the internet environment, the multidimensional collaborative law of environmental economy is studied by using the qualitative analysis method, and the mechanism of environmental collaborative management of circular economy and the standard system of service quality evaluation are put forward. By adjusting the order parameter, the system balance can be effectively controlled and the uncertainty of key factors of environmental economic system synergy of environmental economic enterprises can be effectively solved. At the same time, the case analysis method is adopted to solve the problems of strategic management coordination, distribution management coordination, service management coordination, and warehouse management coordination in the technology, information, service, and management coordination of environmental economic enterprises at the four levels of perception, network, application, and management. The reasonable application of the internet-of-things technology in collaborative management of environment and economy has been solved.

## 3. Multidimensional Collaborative Management Framework of Environment and Economy Based on Internet of Things

### 3.1. Multidimensional Collaborative Management Model of Environment and Economy

Multidimensional environmental economic integration is the environmental economy and adverse environment, which not only includes waste product recycling, classification, detection, and dismantling of processing and remanufacturing reverse environmental economic process but also includes new products and remanufacturing product warehousing, distribution, and distribution of positive environmental economic process, and the network structure is complex, which involves many links. So, full use of the internet of things, cloud computing, big data, and other information and communication technology should be made, for the system in different regions and different nodes, different functions of enterprises should be assumed with information sharing and interaction platform, the remanufacturing environmental economic tasks, processes, and resources for collaborative management, multidimensional environmental economic intelligent decision should be implemented, and control is particularly important. On the one hand, collaborative management module is the source of information and data for remanufacturing environmental economy to realize information synergy, and it is also the specific object and target of the practical application of results of information synergy. Therefore, collaborative management module is the foundation and core of multidimensional environmental economic information synergy. As shown in Figure 1, the architecture is based on three-layer architecture of internet of things, and the information contained in the multidimensional environmental economic coordinated management, match, management, decision management, and collaborative management four-function modules, according to the information service level, can be divided into resource integration, perceptual recognition, data transmission, information integration, and application service in five parts.

The article "Multidimensional Collaborative Management of Environment and Economy in the Internet-of-Things Environment" was retracted in 2023. Reasons: unreliable results or conclusions; concerns about the data; concerns about the peer review; concerns about the citations.

Resource integration is mainly on the dimensional environmental economic participation in enterprise, or the key nodes have, or involved in plant, equipment, distribution transport vehicles, storage space, and remanufacturing of auto parts and other physical resources are classified and integrated, at the same time on the physical properties of various kinds of resources and the classification characteristics of information coding and classification, in order to be equipped with perception and transmission components. It provides material basis for the internet of things to perceive and recognize objects and collect data and information. Perception recognition refers to remanufacturing infrastructure, production equipment, and transportation equipment physical resources such as all kinds of radio frequency identification devices, sensors, global positioning system (GPS), and wireless sensor networks, and the dimensional environmental physical quantity in physical resources of the economy, such as chemical content, and biomass is converted into digital signals, related processing, and communication task. In this way, the dynamic perception and recognition of physical manufacturing resources can be realized, and the requirements of real-time and accurate information acquisition for remanufacturing information coordination can be met.

Data information and control information can be transmitted bidirectionally and shared interactively. Information integration is based on cloud computing, cloud storage, virtualization technology, and database knowledge discovery technology of distributed processing and distributed database support, through the mass data storage, parallel computing and data mining, complete intelligent massive data processing, integration of multisource heterogeneous processing of sensory information, and meets the demand of multidimensional environmental coordinated economic management information. Application service is based on service-oriented architecture, through the cloud computing, big data, fuzzy identification of intelligent computing technology, such as building multidimensional environmental economic key links and different business needs of the system software service platform, and the application of different function modular, and the coordinated management of multidimensional environmental economic information fast and repeatable development and deployment is realized.

The article "Multidimensional Collaborative Management of Environment and Economy in the Internet-of-Things Environment" was retracted in 2023. Reasons: unreliable results or conclusions; concerns about the data; concerns about the peer review; concerns about the citations.

### 3.2. Establishment and Solution of Multidimensional Environmental Economic Synergetic Order Parameter Equation

The system synergetic efficiency is set as Y, the service synergetic factor is set as *x*, as a function of time *t*, the system initial state synergy efficiency is set as Y0, and the balanced synergy efficiency is set as Y:

(1) $$\begin{array}{c} Y=\left\{\begin{array}{c} Y0,\\ \alpha X.\\ Y_{i}.s \end{array}\right) \end{array}$$

System synergetic efficiency is set as S, management synergy factor is set as *T*, and S is a function of *T*.

(2) $$\begin{array}{c} S\left(\partial \right)=\left\{\begin{array}{c} S0,\\ \alpha \chi +S0,\\ S_{i}. \end{array}\right) \end{array}$$

For the complex multidimensional environmental and economic cooperative management system, the macroscopic changes of the system do not depend on the forced action of a given external force but on the “synergy” of subsystems. Whether it is technology synergy, service synergy, or management synergy, they all depend on information synergy and affect the efficiency of information synergy. The modern multidimensional environmental and economic collaborative management information collaborative system can be described by the following equation:

(3) $$\begin{array}{c} \frac{{\text{d}}_{q}}{{\text{d}}_{t}}=\ln\left(q+a\right)+a_{1}q_{1}. \end{array}$$

The synergetic state of the system is shown in Figure 2. By controlling the system order parameters, the synergetic state of the system can be maintained within a certain stable range.

### 3.3. Construction and Key Links of Multidimensional Environmental and Economic Cooperation Model

In the internet-of-things environment, guided by the idea of collaborative management and combined with the requirements of multidimensional environmental and economic management, a comprehensive collaborative model of multidimensional environment and economy is designed to achieve intensive and lean management of multidimensional environment and economy, as shown in Figure 3.

Business process is mainly the sequence from the planning and design stage to the next updated stage according to time, and its core is the process of system operation and implementation in the whole process of the project. The closed-loop management of the whole process is the optimization and improvement of the existing business process and an important element of lean management. As a basic element of asset collaborative management, business process collaboration needs to be comprehensively examined and optimized to improve the existing business process so as to achieve the fundamental improvement of cost, quality, and efficiency. The collaborative process system takes the core business of multidimensional environmental economy as the main line and carries on the collaborative optimization of business processes from the perspective of multidimensional environmental economy. We standardize and coordinate material management from the source of multidimensional environmental economy to ensure smooth connection of business processes until the end of multidimensional environmental economy, and improve the business connection and information transmission of reverse multidimensional environmental economic coordination management and demand planning management.

The article "Multidimensional Collaborative Management of Environment and Economy in the Internet-of-Things Environment" was retracted in 2023. Reasons: unreliable results or conclusions; concerns about the data; concerns about the peer review; concerns about the citations.

According to the conditions a for the existence of extreme values *d*, it can be obtained the following:

(4) $$\begin{array}{c} \frac{\partial S}{\partial x}=\alpha x-\beta \frac{\sum d\left(x_{i},x_{l}\right)}{\max\sum d\left(x_{i},x_{l}\right)}+\lambda . \end{array}$$

The coordination ability of the ethical system of multidimensional environmental economic ethics under the existing constitutional order and code of conduct is determined by what specific operating rules are formulated. The impact of the new institutional arrangement on the multidimensional environment, economic costs, interest relations among stakeholders and the allocation efficiency of internal shared resources.  Table 1 lists the analytical framework for demand and supply of institutional arrangements.

According to the principle of benefit maximization, multidimensional environmental economy decides system coordination supply, adjusts economic policy, formulates new rules or conditions, and establishes a new behavior constraint mechanism. In order to reduce the resistance of multidimensional environmental economy to the implementation of new rules and reduce the transaction costs and management costs within the organization, the member enterprises should unify their ideas and establish a set of ideology and group culture that can be accepted by all the member enterprises in the organization.

One type of institutional synergy is mandatory institutional synergy, which is actually a supply-led institutional synergy. In other words, under certain constitutional procedures and behavioral ethics, the ability and willingness of the power center to provide new institutional arrangements are the leading factors determining institutional synergy. This ability and willingness are mainly determined by the power structure or power balance of various vested interest groups in a society. In the social game in which government and nongovernment subjects participate in the multidimensional environmental and economic system arrangement, government subjects are in a dominant position in the comparison of political forces and the power of resource allocation.

The article "Multidimensional Collaborative Management of Environment and Economy in the Internet-of-Things Environment" was retracted in 2023. Reasons: unreliable results or conclusions; concerns about the data; concerns about the peer review; concerns about the citations.

*Pan* at the location sensing layer is based on the vehicle or handheld mobile intelligent terminals, the embedded vehicle identification device, perception, and two-mode organic fusion of satellite positioning system, through the front-end multidimensional environment economic vehicle intelligent terminal of cooperative management, and all kinds of smart sensors, GPRS/GPS module, and effective integration of front vehicle control together realize real-time perception recognition and effective return control of multidimensional environmental and economic cooperative management vehicles. At the same time, the front-end positioning perception system is integrated with the intelligent multidimensional environmental economic collaborative management terminal system and intelligent multidimensional environmental economic collaborative management service system. It can complete basic information management, vehicle and driver multidimensional environmental economic coordinated management, and distribution system of statistics and management of the day-to-day business, multidimensional environmental economic coordination of the vehicle network management system of unified scheduling, and the whole system maintenance, such as functions, and thus realize the coordinated management of remanufacturing multidimensional environmental economic distribution system visualization and transparent. *Pan* in the location sensing support layer will mainly pan in the location sensing layer under different formats and different identity system provided by ZhiNengDuo dimension of environmental economic coordinated management and distribution service system and environmental ZhiNengDuo dimensions of economic coordinated management and distribution terminal system, and provided across different identity system is the goal of addressing and resolution, and across different positioning system clock synchronization and the coordinate transformation. In this way, the application layer of intelligent multidimensional environmental economic collaborative management and distribution service can eliminate the influence of different standards and different labeling systems, and realize cross-network and cross-system access to intelligent multidimensional environmental economic collaborative management service system and intelligent multidimensional environmental economic collaborative management terminal system, see Figure 4.

Multidimensional collaborative management of environment and economy of intelligent distribution application layer locates the distributed materials or products through RFID (radio frequency identification) perception recognition technology, the in-vehicle terminals with GPS (global positioning system) dual-positioning engines locate the distribution vehicles in operation, and the people involved in multidimensional collaborative management of environment and economy and distribution through handheld mobile intelligent terminals. The combination of these three intelligent application form under the environment of internet of things dimension of environmental economic coordination management in location-aware system, realize the people/car/real-time positioning, real-time tracking, through flexible scheduling staff, and allocate vehicles and goods, to ensure timely response and feedback, vehicles, and supplies safe and controllable. Finally, the utilization efficiency of remanufacturing multidimensional environmental and economic collaborative management and distribution resources is maximized.

The article "Multidimensional Collaborative Management of Environment and Economy in the Internet-of-Things Environment" was retracted in 2023. Reasons: unreliable results or conclusions; concerns about the data; concerns about the peer review; concerns about the citations.

## 4. Results and Analysis

MATLAB was used to calculate, and a 200d dataset of 100 mobile nodes was constructed in the selected area of the case.

**Experiment 1 .**

The construction of condensed subgroups of mobile multidimensional environmental and economic collaborative management service nodes. By calculating the social relation matrix *M* of 100 mobile nodes, the clustering experiment result graph was obtained, see Figure 5.

Mobile multidimensional environmental and economic collaborative management service nodes are clustered according to social relations to form condensed subgroups with special network characteristics. For example, some aggregation subgroups take a large number of sending service requests as the aggregation factor and concentrate in a specific area. Taking campus as an example, the office area is a region with relatively intensive sending and receiving requests for mobile multidimensional environment and economic collaborative management service. Therefore, when setting up multidimensional environmental and economic collaborative management distribution transfer stations, the number and location of distribution personnel, more stations, and staff should be set up in areas with intensive service requests for multidimensional environmental and economic collaborative management, so as to meet a large number of multidimensional environmental and economic collaborative management service demands. Compared with office area, there are relatively few mobile multidimensional collaborative management service nodes of environment and economy in living area. Service quality and operation efficiency are improved according to mobile node clustering.

The article "Multidimensional Collaborative Management of Environment and Economy in the Internet-of-Things Environment" was retracted in 2023. Reasons: unreliable results or conclusions; concerns about the data; concerns about the peer review; concerns about the citations.

**Experiment 2 .**

Moving the shortest distance of multidimensional environmental and economic collaborative management service node.

The shortest distance between mobile nodes and the average distance of the network were analyzed. Three condensed subgroup networks in experimental result 1 were selected for analysis and network parity distance. The experimental results are shown in Figure 6.

The experimental results verify that the shortest distance between nodes and the average distance of the whole network decrease with the increasing complexity of the social relations of the mobile multidimensional environmental and economic collaborative management service nodes. The reduction in the average distance of the network can significantly improve the corresponding efficiency of mobile multidimensional environmental and economic collaborative management service requests, that is, when the interaction and perception between nodes in the network and between nodes in the network are closer, the perception and discovery of multidimensional environmental and economic collaborative management service are more effective.

**Experiment 3 .**

Efficiency of multidimensional environmental and economic collaborative management perceptive service node discovery algorithm.

When the number of mobile nodes ranged from 5 to 40 and the search times is 50, the search success rate of mobile notification service node was calculated. The experimental results are shown in Figure 7.

The experimental results show that with the increase in the number of mobile multidimensional environmental and economic collaborative management service nodes, the network density begins to increase, and the location information of nodes becomes more complex, which makes the success rate of service node perception continuously improve.

In order to verify the effectiveness of the cooperative model of multistage inventory in remanufacturing, the example in this section assigns values to all parameters of the model, uses numerical simulation to find the optimal solution of the model, and then analyzes and compares the total profit of the whole system under the conditions of cooperative decision-making and independent decision-making.

The specific values assigned to each parameter of the inventory synergy model are shown in Table 2:

The above parameter values were substituted into the corresponding formula of the model and solved by MATLAB. The optimal solution obtained is shown in Table 3.

From the result, it is shown that the enterprise collaborative management members take multidimensional environmental economic coordinated decision under the condition of the whole system of the gross profit was 169478, more than individual decisions' profit increased by 7.15%, namely, dimensional environmental economic coordinated management takes multilevel inventory decisions that can effectively reduce the inventory cost, improve the system as a whole the profits of the water, and bring more profit for the whole multidimensional environmental and economic cooperative management system.

The article "Multidimensional Collaborative Management of Environment and Economy in the Internet-of-Things Environment" was retracted in 2023. Reasons: unreliable results or conclusions; concerns about the data; concerns about the peer review; concerns about the citations.

By comparing the profits of distributors, manufacturers/remanufacturers, recyclers, and suppliers under cooperative decision and independent decision in multidimensional environmental and economic cooperative management, it is found that in the same cycle, except that the profit level of distributors slightly decreases under cooperative decision. Other multidimensional collaborative management of environment and economy can increase profits for enterprises by adopting inventory collaborative decision.

In order to reflect the advantages and practicability of the internal and external information collaborative simulation of the distribution module, the dynamic information and the traditional static information considering the multidimensional environmental and economic collaborative management were simulated, respectively, and the simulation results were verified and compared. Its simulation data are shown in Figure 8.

Because the traditional simulation method takes distance as the optimization target and does not consider the cooperative management information, it cannot make real-time response to the multidimensional environmental and economic cooperative management, and the path distance length does not significantly change. In the simulation of information collaboration, information managed by the internet of things will be selected in the case of coordination and management, as shown in Figure 9.

Due to the historical regularity of various traffic behaviors in a day, the coordinated management of multidimensional environment and economy is different in different time periods in the city. Therefore, the start time of distribution also affects the overall effect of distribution. The number of urban nodes is set as 10, and the original speed of distribution vehicles is set as 200. The experimental results are shown in the figure below. In the traditional simulation process, the whole time in the simulation results is longer than that in the information cosimulation because coordination management is only taken as the objective of optimization, so the optimal path cannot be found, see Figure 10.

We must speed up the construction of market organization and market mechanism while pushing the multidimensional environmental and economic coordinated management into the market. In this regard, there are three basic conditions: first, to improve the factor market system, including capital market, labor market, technology market, and information market, so that inputs can freely flow within the social scope, which is a necessary condition for promoting the coordinated management of multidimensional environment and economy to the market. Second is the perfect price system. Price is a function of market supply and demand, and the result of negotiation between buyers and sellers in market competition on the basis of possessing the same information. Therefore, the determination of prices according to the same market rules is the basis of market structure. Third, market rules should be improved. Whether it is the traditional market trading rules or the modern market rules established by government authority and legal norms, the simplification and standardization of the rules are the basis for the effective operation of the market.

The article "Multidimensional Collaborative Management of Environment and Economy in the Internet-of-Things Environment" was retracted in 2023. Reasons: unreliable results or conclusions; concerns about the data; concerns about the peer review; concerns about the citations.

## 5. Conclusions

The multidimensional environmental economic cooperation management based on capital is the foundation of establishing modern enterprise system. In the process of carrying out the coordinated management of large-scale and multidimensional environmental economy in China, in order to realize the organic combination of extension expansion and internal innovation, we should take the modern enterprise system as the direction, and the multidimensional environmental economy in collaborative management should take the lead in establishing the modern enterprise system so as to realize the high-efficiency operation of the group. In view of the problems faced by multidimensional environmental and economic collaborative management enterprises, the multidimensional collaborative classification of the modern multidimensional environmental and economic collaborative management is proposed. In this study, the multidimensional collaborative order parameter equation of the modern multidimensional environmental and economic collaborative management system is constructed, and the information synergy is the order parameter of the multidimensional environmental and economic collaborative management system, and the fluctuation and balance of the multidimensional environmental and economic collaborative management system are accurately controlled by the order parameter. The multiagent collaborative model of the modern multidimensional environmental and economic collaborative management of internet-of-things network layer under cooperative game is proposed. Aiming at the collaborative problem of multidimensional environmental and economic collaborative management of enterprise distribution management, a real-time road condition information collaborative simulation model based on VRP is constructed. Through simulation and numerical experiment, it is proved that information synergy can obviously improve the efficiency of multidimensional environmental and economic cooperative management system. In view of the research on information coordination of multidimensional environmental and economic system based on the internet of things, due to the limitation of technology, only the commonness of environmental and economic industries is considered, and the differences in different industries are not analyzed and discussed.

The article "Multidimensional Collaborative Management of Environment and Economy in the Internet-of-Things Environment" was retracted in 2023. Reasons: unreliable results or conclusions; concerns about the data; concerns about the peer review; concerns about the citations.

## Figures and Tables

**Figure 1:** Overall architecture of multidimensional environmental and economic information coordination based on internet of things.

**Figure 2:** Synergistic superposition of multidimensional environment and economy.

**Figure 3:** Multidimensional collaborative model of environmental economy.

**Figure 4:** Ubiquitous positioning system architecture for collaborative management of intelligent multidimensional environment and economy.

**Figure 5:** Division of condensed subgroups of mobile multidimensional environmental and economic collaborative management service node network.

**Figure 6:** Distance analysis of mobile multidimensional environmental and economic collaborative management service nodes.

**Figure 7:** The number of mobile multidimensional environmental and economic collaborative management service nodes.

**Figure 8:** Multidimensional collaborative management of environment and economy.

**Figure 9:** Analysis and comparison of multidimensional environmental and economic collaborative management.

**Figure 10:** Effect diagram of multidimensional collaborative management of environment and economy in the internet-of-things environment.

**Table 1:** Overview of the analytical framework for demand and supply of institutional arrangements.

System category	Endogenous variables	Exogenous variables of the need for institutional change	Exogenous variables: the supply of institutional change	Dynamic order
Constitutional order institutional arrangement normative code of conduct.	Institutional arrangements: the extent to which institutional arrangements are utilized.	Relative products and elements price (including demographic change): constitutional order: technology: market size.	Constitutional order: existing institutional arrangements: cost of institutional design: now knowledge accumulation: expected costs of implementing the new arrangements: normative code of conduct: public attitude: the expected benefits of top decision-makers.	Change means institutional evolution.

**Table 2:** Model parameter assignment list.

Name of the parameter	Parameter value
Manufacturer's output of new products per unit cycle	Article 6000/month
Unit cycle manufacturer remanufacturing product output	Article 4000/month
Finished goods purchased by distributor per unit cycle	Article 12000/month
Purchasing raw materials from suppliers per unit cycle	2600 tons

The article "Multidimensional Collaborative Management of Environment and Economy in the Internet-of-Things Environment" was retracted in 2023. Reasons: unreliable results or conclusions; concerns about the data; concerns about the peer review; concerns about the citations.

**Table 3:** Solutions of collaborative management model of internet-of-things environment and economy.

Model variables	K (key)	T (time)	Q (query)	M (varia)	N (varia)	TPt	TPq	TPm	Jp
Coordination decision	4	5	930	320	5	41231	24389	35793	169478
Independent decisions	6	8	1240	632	9	42391	20492	30573	157834

## Data Availability

The data used to support the findings of this study are available from the corresponding author upon request.
